RETRACTED

# Basketball Sports Injury Prediction Model Based on the Grey Theory Neural Network

**DOI:** 10.1155/2021/1653093

**Published:** 2021-08-21

**Authors:** Fengyan Zhang, Ying Huang, Wengang Ren

**Affiliations:** ^1^Physical Education Department, Shijiazhuang Information Engineering Vocational College, Shijiazhuang 05000, Hebei, China; ^2^Department of Sports Arts, Hebei Sport University, Shijiazhuang 05000, Hebei, China; ^3^Department of Sports Training, Hebei Sport University, Shijiazhuang 05000, Hebei, China

## Abstract

Sports injuries will have an impact on the consistency and systemicity of the training process, as well as athlete training and performance improvement. Many talented athletes have had their careers cut short due to sports injuries. Preventing sports injuries is the best way for basketball players to reduce sports injuries. Many coaches and athletes on sports teams, on the other hand, are unaware of the importance of sports injury prevention. They only realize that the body's sports functions are abnormal when it suffers from sports injuries. As a result, this paper proposes a gray theory neural network-based athlete injury prediction model. First, from the standpoint of a single model, the improved unequal interval model is used to predict sports injury by optimizing the unequal interval model in gray theory. The findings show that it is a good predictor of sports injuries, but it is a poor predictor of the average number of injuries. Following that, in order to overcome the shortcomings of a single model, a gray neural network combination model was used. A combination model of the unequal time interval model and BP neural network was determined and established. The prediction effect is significantly improved by combining the gray neural network mapping model and the coupling model to predict the two characteristics of sports injuries. Finally, simulation experiments show that the proposed method is effective.

## 1. Introduction

The pursuit of a healthy life has become a goal for modern people as their quality of life has improved. For today's people, a healthy diet and regular exercise have become a common way of maintaining their health [1–3]. Regular exercise can help people improve their physical fitness by improving various body functions and recognize the benefits of body strengthening. Sports, on the other hand, come with varying degrees of risk. Many people lack a basic understanding of various sports, and their personal circumstances do not meet the requirements for completing a sport [4, 5], resulting in varying degrees of injury [6, 7]. Not only do they fail to strengthen their bodies but also in severe cases, it can cause long-term damage and even life threatening. In competitive training [8–10], competitions and fitness sports, insufficient preparation, improper training, technical errors, etc. are also the main causes of sports injuries [11, 12].

RETRACTED

Basketball is a highly antagonistic open sport that necessitates a high level of physical fitness. The gradual acceleration of the game rhythm, the more intense physical confrontation of athletes, and the continuous improvement of athletes' outside shooting ability are all examples of modern basketball style. Athletes must have a higher level of physical fitness, technical proficiency, and the ability to use techniques and tactics. The speed of competition continues to increase as the level of Cuba athletes' sports improves, and the physical confrontation becomes more fierce [13, 14]. At the same time, the number of basketball players who sustain sports injuries is on the rise [14, 15]. Basketball is also considered a high-intensity sports event in terms of injuries. The continuity of an athlete's training process and the systemicity of the training plan will be shattered if the athlete sustains a sports injury. It will also have an impact on the athlete's competitive state and hinder their progress in sports. A serious sports injury can even put an athlete's career on hold. The majority of CU basketball players lack basic theoretical knowledge of sports injuries, pay little attention to sports injuries, and are unaware of how to prevent sports injuries [16, 17]. Many athletes only find abnormalities in physical function when sports injuries occur. If you want to reduce sports injuries, in fact, the best way is to prevent the occurrence of sports injuries.

Through investigation, this article found that some existing studies on the causes, types, and measures of sports injuries are relatively shallow, insufficiently in-depth, relatively limited, and have more blind spots. Therefore, the purpose of this article is to understand and study basketball players. The rules and characteristics of sports injuries are as follows. The investigation's goal is to protect athletes from injury and provide references for coaches in the process of coaching and training teams [18], as well as to implement targeted preventive measures during training and competitions to provide athletes with sports injury prevention and reduction. The corresponding reference is to raise awareness of the importance of sports injuries among coaches and athletes, as well as the measures and methods for dealing with them. Effective training methods are used and explored, and corresponding suggestions and methods are provided for basketball players to prevent sports injuries, in order to meet the needs of athletes to reduce sports injuries and improve sports performance.

RETRACTED

At present, a lot of artificial intelligence technologies have been applied in the field of health, such as image processing [19, 20] and medical single processing [21, 22]. Therefore, this paper proposes an athlete injury prediction model [23] based on gray theory [24–26] and neural network technologies [27, 28]. First, from the perspective of a single model, by optimizing the unequal interval model in gray theory, the improved unequal interval model is used to predict sports injury. The results show that it has a good predictive ability for sports injuries, but it has a poor predictive effect on the average number of injuries. Subsequently, in order to overcome the shortcomings of a single model, a combination model of gray neural network [29, 30] was adopted. We determined and established a combination model of the unequal time interval model and BP neural network. With the comprehensive use of the gray neural network mapping model and coupling model to predict the two characteristics of sports injuries, the prediction effect is significantly improved. Finally, simulation experiments prove the effectiveness of the proposed method.

Following are the main innovations of this paper:

1. In this paper, by optimizing the unequal interval model in gray theory, the improved unequal interval model is used to predict sports injuries, which improves the prediction ability. Secondly, in order to overcome the shortcomings of a single model, we establish a combination model of the unequal interval model and BP neural network.
2. In this paper, a combination of the gray neural network mapping model and coupling model is used to predict the two characteristics of sports injuries, and the prediction effect is significantly improved. Finally, simulation experiments prove the effectiveness of the proposed method.

## 2. Background

Basketball is a team sport with a large number of players and intense physical competition. During competition and training, basketball players must engage in intense physical contact and physical confrontation, as well as various acceleration and emergency stop actions. During the course of these sports, various parts of the body are prone to sports injuries as a result of sharp turns, jumps, and landings during fierce confrontations. Basketball sports injuries and prevention has been the subject of numerous domestic and international studies.

Some scholars have analyzed the mechanism theory of the joint injury of amateur college basketball players from an anatomical point of view. Researchers believe that according to the physiological characteristics of the human anatomy, the ankle, knee, and lumbar joints are more likely to be injured in basketball. It is believed that basketball players should increase their awareness of preventing sports injuries psychologically, perform adequate preparation activities before basketball games, strengthen the training of muscles around the joints that are prone to damage during training, enhance the athletic ability of related muscles, and strengthen medical supervision. Also, the inspection and maintenance of stadium equipment shoyld be carried out.

RETRACTED

Basketball sport injury rate is higher, and the scholars, mainly from the athletes for the understanding of the knowledge of basketball sports injury degree, sports injury, sports injury type, nature of the sports injury, sports injury situation and causes of sports injury, and sports injury prevention, research basketball sports injury and ankle and knee injury mainly; the main types of injury were sprain and strain. Injury nature acute injury is more; most of the injuries were caused during training. Causes of injury: biological factors are mainly due to the unique technical movements of basketball and the special anatomical structure of the knee joint. Other training learning factors include insufficient physical quality, with training, no timely recovery, basketball basic technical movements that are not standard, the local burden, no timely treatment, the body fatigue, adjusting the unreasonable, insufficient attention to prepare activity and relaxation stretching, inattention, training system, excessive excitement, and depression. In terms of basketball injury prevention, effective prevention methods are insufficient, athletes' awareness of injury prevention is insufficient, ability is insufficient, and self-protection awareness must be improved.

Most researchers believe that the most effective way to prevent basketball sports injuries is to use scientific, reasonable, and effective training methods to improve athletes' body movement ability in order to achieve the goal of sports injury prevention, strengthen the body's own protection ability, and so on for the prevention of basketball injuries and the rehabilitation of research. Lack of knowledge of basketball sports injury and rehabilitation training methods should raise awareness among basketball coaches and athletes to prevent sports injury, allowing them to master more knowledge of basketball sports injury and rehabilitation training methods, allowing them to effectively prevent basketball athlete sports injury and extend their sports careers. According to the research in recent years, some scholars believe that the athletes' sports injury because of motor movements with defects, motion compensation, and the body appeared about asymmetrically because that would lead to the drop in target action sports ability, insufficient muscle strength, and the adjacent joint and muscle motion compensation, and the whole body movement function chain is destroyed. The ability to exercise is limited, which leads to an increased risk of sports injuries.

RETRACTED

## 3. Methodology

### 3.1. Research Object

Table 1 shows the basic information of the four women's basketball teams tested. According to their basic information, most of them are between 19 and 23 years of age. The youngest player from university A is only 18 years old, while the oldest player from university B is 25 years old, which is also the upper age limit stipulated by the Cuba Chinese University Basketball League. Players from university C and university A are relatively young. The players of university D are weaker than those of the other three teams in terms of weight. The heaviest and lightest players are from university A, while the height of players of university C is lower than those of the other three teams. The tallest and shortest players are also from university A, 1.63 meters and 1.92 meters, respectively. The 45 participants were 20.98 ± 1.41 years old, 1.78 ± 0.06 meters in height, and 70.80 ± 11.84 kg in weight.

### 3.2. Grey Prediction Model

#### 3.2.1. Grey Sequence Generation

The main idea of gray theory is to find out its own mathematical relationship and development and change rules by analyzing the behavior data of the target. We set the time series *x*^(0)^ as *n* nonnegative original observation values:

(1) $$\begin{array}{c} x^{\left(0\right)}=\left\{x^{\left(0\right)}\left(1\right),x^{\left(0\right)}\left(2\right),\ldots ,x^{\left(0\right)}\left(n\right)\right\}. \end{array}$$

We perform a quasismoothness test on *x*^(0)^ and set *σ*(*k*)=(*x*(*k*)/*x*(*k* − 1)),  *k*=2,3,…, *n* as the original sequence ratio. *ρ*(*k*)=(*x*(*k*)/∑_*i*−1_^*k*−1^*x*(*i*)),  *k*=2,3,…, *n* is the smooth ratio of the original sequence.

When the original sequence meets the inspection requirements, gray theory can be used for modeling. First, 1-AGO (Acumulated Generating Operator) first-order accumulation is used to reduce the randomness of the original sequence and enhance the regularity to a certain extent.

Definition: we perform 1-AGO on the original data *x*^(0)^ to generate a sequence:

(2) $$\begin{array}{c} x^{\left(1\right)}=\left\{x^{\left(1\right)}\left(1\right),x^{\left(1\right)}\left(2\right),\ldots ,x^{\left(1\right)}\left(n\right)\right\},\\ x^{\left(1\right)}\left(1\right)=\sum_{i-1}^{k}x^{\left(0\right)}\left(i\right),\;k=1,2,\ldots ,n. \end{array}$$

We determine the GM (1,1) model and establish the whitening equation:

(3) $$\begin{array}{c} \frac{\text{d}x^{\left(1\right)}}{\text{d}t}+ax^{\left(1\right)}=b, \end{array}$$

where *a* is called the development coefficient, which represents the speed of change of the original sequence; *b* is called the gray effect, which represents the relationship between the data. We discretize the abovementioned formula to get the GM (1, 1) gray differential equation:

(4) $$\begin{array}{c} x^{\left(0\right)}\left(k\right)=az^{\left(1\right)}\left(k\right)=b,\;k=1,2,\ldots ,n, \end{array}$$

where *z*^(1)^={*z*^(1)^(1), *z*^(1)^(2),…, *z*^(1)^(*n*)} is used as the next-generation sequence of *x*^(1)^, which is called the gray model background value.

(5) $$\begin{array}{c} z^{\left(1\right)}=\frac{1}{2}\left[x^{\left(1\right)}\left(k-1\right)+x^{\left(1\right)}\left(k\right)\right],\;k=1,2,\ldots ,n. \end{array}$$

According to the principle of least squares method, the characteristic parameters in the gray differential equation are solved, and the result is

(6) $$\begin{array}{c} {\left(\hat{a},\hat{b}\right)}^{T}={\left(B^{T}B\right)}^{-1}B^{T}Y, \end{array}$$

where

(7) $$\begin{array}{c} B=\left[\begin{array}{cc} -z^{\left(1\right)}\left(2\right) & 1\\ -z^{\left(1\right)}\left(3\right) & 1\\ \vdots & \vdots \\ -z^{\left(1\right)}\left(n\right) & 1 \end{array}\right],\\ Y=\left[x^{\left(0\right)}\left(2\right),x^{\left(0\right)}\left(3\right),\ldots ,x^{\left(0\right)}\left(n\right)\right]. \end{array}$$

Substituting the characteristic parameters into the gray differential equation, the time response sequence of GM (1,1) is obtained as

(8) $$\begin{array}{c} {\hat{x}}^{\left(1\right)}\left(k+1\right)=\left(x^{\left(1\right)}\left(0\right)-\frac{b}{a}\right)e^{-ak}+\frac{b}{a},\;k=1,2,\ldots ,n. \end{array}$$

We take *x*^(1)^(0)=*x*^(0)^(1):

(9) $$\begin{array}{c} {\hat{x}}^{\left(1\right)}\left(k+1\right)=\left(x^{\left(0\right)}\left(1\right)-\frac{b}{a}\right)e^{-ak}+\frac{b}{a},\;k=1,2,\ldots ,n. \end{array}$$

We restore the result value to get the original sequence prediction value:

(10) $$\begin{array}{c} {\hat{x}}^{\left(0\right)}\left(k+1\right)={\hat{x}}^{\left(1\right)}\left(k+1\right)-{\hat{x}}^{\left(1\right)}\left(k\right),\;k=1,2,\ldots ,n. \end{array}$$

RETRACTED

#### 3.2.2. Model Test

Whether a forecasting model is suitable for related problems after it is established, the model's credibility must be tested before the results can be effectively applied in the actual forecasting process. Postevent prediction and preprediction are two commonly used test methods for predictive models. The postevent prediction is based primarily on data that have already occurred; the preprediction is a prediction of what will occur but has yet to occur. As a result, as shown in Figure 1, two inspection ideas are used in the actual forecasting work.

The grey correlation test is one of the accuracy test methods that are part of gray theory. After the prediction model is established, the relevance test is used to determine how close the predicted sequence is to the original sequence, and the degree of relevance is determined by comparing the geometric shape of the data curve. The higher the degree of association, the closer the data graph's change trend. The degree of association, on the other hand, is minimal. We assume the following sequence:

(11) $$\begin{array}{c} x_{0}^{\left(0\right)}=\left[x^{\left(0\right)}\left(1\right),x^{\left(0\right)}\left(2\right),\ldots ,x^{\left(0\right)}\left(n\right)\right]. \end{array}$$

The forecast sequence is

(12) $$\begin{array}{c} {\hat{x}}_{i}^{\left(0\right)}=\left[{\hat{x}}^{\left(0\right)}\left(1\right),{\hat{x}}^{\left(0\right)}\left(2\right),\ldots ,{\hat{x}}^{\left(0\right)}\left(n\right)\right]. \end{array}$$

Then, the degree of relevance is

(13) $$\begin{array}{c} \delta_{i}\left(k\right)=\frac{\underset{i}{\min}\underset{k}{\min}\left|{\hat{x}}_{i}\left(k\right)-x_{0}\left(k\right)\right|+\rho \underset{i}{\min}\underset{i}{\min}\left|{\hat{x}}_{i}\left(k\right)-x_{0}\left(k\right)\right|}{\left|{\hat{x}}_{i}\left(k\right)-x_{0}\left(k\right)\right|+\rho \underset{i}{\min}\underset{i}{\min}\left|{\hat{x}}_{i}\left(k\right)-x_{0}\left(k\right)\right|}, \end{array}$$

where *ρ* is called the resolution coefficient and usually takes the value *ρ*=0.5. So, the degree of correlation between sequences is

(14) $$\begin{array}{c} \delta \left(k\right)=\frac{1}{n}\sum_{k=1}^{n}\delta_{i}\left(k\right). \end{array}$$

### 3.3. Grey Neural Network

So far, the research of gray neural network combination has made great progress, and good results have been achieved in different fields. The common structures are series and coupling types, as shown in Figure 2.

The series structure is to connect the gray model with the neural network; that is, the output of one side is the input of the other side, including residual correction and neural network weighted prediction of multiple gray models.

The coupled structure makes full use of the gray theory's data processing capabilities for sample objects, and ashing the samples weakens the randomness of the original samples. The ashing layer processes the original data, which are often generated by first-order accumulation or accumulation. We put the ashed samples into the neural network for training and use the self-learning ability of the neural network to improve the prediction accuracy. The ashed samples are conducive to network convergence, shortening the learning time and reducing the requirements for the number of samples, as shown in Figure 3.

RETRACTED

## 4. Experiments and Results

### 4.1. Experimental Setup

All experiments of this stability are carried out on a PC, the operating system is Windows 10, the CPU is Inter Core i9-9900k, and the GPU is RTX 2080ti with 11G video memory for accelerating model training and testing. The models used are all in Python 3.6 and Tensorflow 1.8.0, implemented under CUDA9.0 and CUDNN 7.1.

### 4.2. Evaluation Index

Relative error (RE) takes the actual value as the reference value and judges by comparing the relative difference between the predicted result of the target data and the actual value. We usually express it as a percentage. The smaller the value of the relative error, the closer the prediction result to the actual value. In other words, the better the prediction effect of the constructed model. Generally speaking, the relative error can better reflect whether the prediction result is credible. The relative error expression is as follows:

(15) $$\begin{array}{c} \text{RE}=\frac{y_{i}-y_{i}^{\prime }}{y_{i}}\times 100\%. \end{array}$$

### 4.3. Experimental Results

A basketball sports injury prediction model is developed using gray theory and neural network analysis of basketball sports injury factors.  Figure 4 depicts the predicted and actual values using the algorithm described in this paper. The blue asterisk in the figure represents the predicted injury value, while the green circle represents the actual number of basketball players injured in the test set.  Figure 4 clearly shows except for a few basketball sports injuries, there is a small difference between the predicted and actual values in the test set. The predicted results of most basketball sports injuries are very close to the actual results. This shows that based on gray theory, the network's basketball injury prediction model is very reliable.

Table 2 is the error analysis and comparison results between the predicted results of basketball sports injuries and the actual results. The relative error of the method in this paper is the lowest. This fully shows that the basketball sports injury prediction model based on the gray theory neural network is very good and the prediction effect of the model is quite satisfactory.

### 4.4. Ablation Experiments

In order to further verify the effectiveness of the algorithm, in this section, an ablation experiment is set up. UI stands for the unequal interval model, improved-UI stands for the improved unequal interval model, CO stands for the coupling model, and GNN stands for the gray neural network.

RETRACTED

It can be seen from Table 3 that the relative error of using the unimproved unequal interval model is the highest. Secondly, although the coupled model can improve the performance of the model to a certain extent, it is still inferior to the model proposed in this paper. This once again proves the effectiveness of our algorithm.

## 5. Conclusions

Sports injuries affect the consistency and systemicity of the training process, as well as the improvement of athletes' training and sports performance, according to this paper. Many talented athletes have had their careers cut short due to sports injuries. Preventing sports injuries is the best way for basketball players to reduce sports injuries. Many coaches and athletes on sports teams, on the other hand, are unaware of the importance of sports injury prevention. They only realize that the body's sports functions are abnormal when it suffers from sports injuries. As a result, this paper proposes a gray theory neural network-based athlete injury prediction model. First, from the standpoint of a single model, the improved unequal interval model is used to predict sports injury by optimizing the unequal interval model in gray theory. The findings show that it is a good predictor of sports injuries, but it is a poor predictor of the average number of injuries. Following that, in order to overcome the shortcomings of the single model, a gray neural network combination model was used. A combination model of unequal time interval model and BP neural network was determined and established. In addition, the results of comparison and ablation experiments prove that the proposed algorithm is competitive.

## Figures and Tables

**Figure 1:** The idea of model test.

**Figure 2:** Tandem structure.

**Figure 3:** Coupled structure.

**Figure 4:** Forecast result.

**Table 1:** Introduction to the GTZAN dataset.

Team	Number of people	Age	Height	Weight
University A	13	19.10	1.69	70.25
University B	10	20.63	1.71	68.22
University C	10	21.25	1.68	60.23
University D	12	22.96	1.60	58.52

**Table 2:** Comparative experiment results.

Method	RE (%)
ARIMA	26
PROPHET	15
BP	12
**Ours**	**9**

**Table 3:** Ablation experiment results.

Method	RE (%)
UI + GNN	16
Improved-UI + GNN	12
UI + CO + GNN	14
**Improved-UI** **+** **CO** **+** **GNN**	**9**

## Data Availability

The data used to support the findings of this study are included within the article.
